# Evaluation of Soluble CD90: Potential for Diagnostic Significance in Endometriosis Patients

**DOI:** 10.1155/2022/9345858

**Published:** 2022-06-20

**Authors:** Ivan M. Bochev, Iliya I. Karagyozov, Nadya M. Magunska, Vesselina S. Koleva, Ivan V. Krumov, Elena S. Puncheva, Georgi P. Boyadzhiev, Kameliya Vinketova, Milena S. Mourdjeva, Tsvetelina P. Oreshkova

**Affiliations:** ^1^Department of Molecular Immunology, Institute of Biology and Immunology of Reproduction, Bulgarian Academy of Sciences, Sofia 1113, Bulgaria; ^2^Ob/Gyn Hospital Dr. Shterev, Sofia 1330, Bulgaria; ^3^Department of Obstetrics and Gynecology, Hospital Vita, Sofia 1407, Bulgaria; ^4^Medical University, Pleven 5800, Bulgaria; ^5^Health Care Department, University of Ruse “Angel Kanchev”, Ruse 7017, Bulgaria; ^6^Clinical Laboratory, Acibadem City Clinic Tokuda Hospital, Sofia 1407, Bulgaria

## Abstract

**Background:**

Endometriosis is a chronic and debilitating gynecologic disorder, driven by endocrine and immune dysfunctions, which lead to poor endometrial differentiation and attenuated fertility. Escape from immune surveillance and involvement of inflammatory mechanisms appear to be factors in disease progression. Current diagnostic guidelines for endometriosis still lack an efficient biomarker. Here, we report a study on two previously unexplored factors as potential biomarkers for endometriosis.

**Methods:**

A case-control study was performed to evaluate the diagnostic potential of serum CD90 and CD83 levels in endometriosis patients (cases validated by surgical and histological examination) compared to healthy controls. Serum was collected from age-matched females and analyzed by ELISA.

**Results:**

Comparison of endometriosis patients to the control group showed significantly elevated levels of serum CD90 (1160 ± 856 pg/mL vs. 334 ± 228 pg/mL; ^∗∗∗∗^*p* < 0.0001). A threshold value of 479.4 pg/mL was defined based on the control results, and the diagnostic efficiency of the test was estimated. The obtained sensitivity (70.4%), specificity (92.9%), positive predictive value (90.5%), and negative predictive value (76.5%) rated the test as one with promising diagnostic potential. In contrast, the analysis of serum CD83 levels showed comparable values in both groups, suggesting no association with patient status.

**Conclusion:**

Elevated soluble CD90 in human serum is associated with endometriosis, which suggests its putative clinical significance as a biomarker in screening and/or diagnosis of the disease.

## 1. Introduction

Endometriosis is a benign, multifactorial gynecologic disease with unclear pathogenesis. It is suggested that genetic [1] and environmental factors interfere in ovarian steroidogenesis and cause the condition [2]. Epidemiology reveals up to 10% prevalence of symptomatic cases in reproductive age women [3]. Endometriosis is diagnosed by visual inspection of lesions in laparoscopy and positive histology of excised tissue [4]. As the diagnosis is invasive and carries risks of postoperative complications [5–7], it is not easily accessible to women who may have the condition. This contributes to the often long delays from onset of symptoms to diagnosis of endometriosis.

Endometriosis manifests with abnormal attachment, invasion, and growth of endometrial stroma and glands in locations outside the uterus. The lesions/implants mainly attach to peritoneal organs [5, 8] but more rarely appear at distant sites, such as the thorax [9, 10]. The lesions exhibit cyclic growth and dominant sensitivity to estrogens [1, 8, 11] but resistance to progesterone [2, 12]. Eutopic endometrial and ectopic endometriosis tissue evades progesterone regulation during the secretory phase of the menstrual cycle. It exhibits impaired proliferation arrest and differentiation of the endometrial stromal cells. The infiltrating immune cells also demonstrate a refractive response to progesterone signaling via NF-*κβ*-mediated proinflammatory activity [13, 14]. The peritoneal lesions evade immune surveillance [11], become refractive to apoptosis, change their adhesive and migratory properties, and produce proinflammatory and oxidative stress molecules [13, 15], which perpetuate an inflammatory environment.

The World Endometriosis Society emphasizes the need for a reliable noninvasive test for endometriosis that could replace the surgical method [6]. A priority of research is discovering measurable marker/s for screening of patients [15, 16] with relevant symptoms, such as abdominal pain and subfertility. So far, no single molecule associated specifically with endometriosis has been identified [3, 16]. As possible markers, immune mediators are of interest because of the inflammatory signature of the disease. This led us to investigate two soluble molecules, CD83 and CD90/Thy-1, which have not yet been tested in connection with endometriosis. They are glycoproteins from the immunoglobulin superfamily that exist in membrane-bound and soluble forms and are involved in fundamental cell processes.

CD90 is a glycosylphosphatidyl inositol-anchored receptor that clusters within lipid raft microdomains in the cell membrane [17]. In humans, CD90 is expressed in neurons, fibroblasts, activated endothelial cells, mesenchymal stem/stromal cells, and multiple cancer types [18], such as brain, kidney, pancreas, liver, and skin tumor cells. It controls stemness, differentiation, migration, survival, and cytoskeleton organization in cells, which are all processes that are affected in endometriosis. At sites of inflammation, activated endothelial cells upregulate CD90 receptor to mediate the extravasation of leukocytes from vessels via *β*_2_ integrins [19]. Using the same mechanism of dissemination, highly invasive tumor cells undergo *α*_v_*β*_3_ integrin-dependent extravasation through CD90-expressing blood and lymphatic vessels [20, 21]. Numerous studies have reported CD90 as a hallmark for cancer stem cells. These cells maintain the growth, invasiveness, and metastatic properties of tumors [22, 23]. Differentiation of tumor stem cells and mesenchymal stromal cells induces decrease of CD90 [22, 24, 25], whereas inflammatory cytokines trigger shedding of CD90 from the membrane of CD90-expressing cells [26]. *In vivo*, soluble CD90 (sCD90) is reported in serum, cerebral spinal fluid, wound fluid, and synovial fluid. Particularly, sCD90 is elevated in patients with systemic sclerosis, venous leg ulcers, and rheumatoid arthritis, with local release from affected tissues [27, 28].

CD83 has regulatory functions, such as activation or suppression of immune cells. The membrane form is a marker for mature dendritic cells [29, 30] but may transiently upregulate in multiple leukocytes at activation [31, 32]. CD83 in DC costimulates T-cells [29, 33] or can suppress the activity of CD83-expressing effector lymphocytes via CD83 homophilic interaction. The soluble form of CD83 (sCD83) has an inhibitory effect on T-cell activation and maturation of dendritic cells [34, 35]. At background level, sCD83 [36] is found in serum and plasma from healthy people and in modified concentrations in patients with hematological malignancies [37], rheumatoid arthritis [38], and juvenile diabetes [39]. Various tumor cell types induce immune suppression via sCD83 release and evade immune surveillance [40, 41].

CD83 and CD90 molecules are associated with cancer and inflammation-mediated diseases. They have a broad spectrum of functions, some of which may hypothetically underlie the inflammatory, invasive, or migratory nature of ectopic endometrium in endometriosis. To explore possible correlations of sCD83 and sCD90 with endometriosis pathophysiology, we measured the molecules in patients' serum in a case-control study.

## 2. Materials and Methods

This study included 57 women (21-46 years) divided into a control group of healthy volunteers (*n* = 30) and an observation group of endometriosis patients (*n* = 27). It was approved by the Bioethics Committee at Acibadem City Clinic Tokuda Hospital, Sofia, and Ob/Gyn Hospital Dr. Shterev, Sofia. All participants signed an informed consent prior to donating peripheral blood to this study. Participants in the control group were in good general health, without symptoms of endometriosis, according to anamnesis. They were also free from acute and chronic diseases or inflammatory conditions.

Endometriosis in patients was diagnosed on the basis of clinical symptoms and examination by sonography, laparoscopy, and histology. The severity of the condition was staged according to the revised classification of the American Society for Reproductive Medicine: I (minimal), II (mild), III (moderate), and IV (severe) [42]. The endometriosis status (staging) and the phase of menstrual cycle of patients are summarized in Table 1. The phase of menstrual cycle of the control group participants was not recorded and is assumed to be random.

Blood samples were collected from the volunteers at the time of their agreement and from the patients with suspected symptoms immediately before the scheduled laparoscopic intervention. The patients had not been previously treated by hormonal medication for endometriosis.

### 2.1. Peripheral Blood Collection and Serum Preparation

Peripheral blood samples were collected from all subjects directly into Vacuette® serum separator tubes (5 mL; Greiner Bio-One) and allowed to clot for two hours at room temperature or overnight at 4°C prior to centrifugation for 20 minutes at 1000 × g at room temperature. The resulting sera were collected, aliquoted, and stored at −20°C for later use.

### 2.2. Enzyme-Linked Immunosorbent Assay

Quantitative measurement of soluble CD90/Thy-1 and CD83 in serum samples was performed using the commercially available ELISA kits of Human Thy1 Cell Surface Antigen (MBS2019822, MyBioSource, Inc.) and Human CD83 Antigen (CD83) (MBS924667, MyBioSource, Inc.) following the instructions provided by the manufacturer. Each serum sample was analyzed in duplicate. In each assay, the absorbance was measured at 450 nm for both molecules and additionally at 544 nm (correction wavelength) for CD83 using a plate reader (FLUOstar OPTIMA, BMG LabTech). The minimum detection limits for the assays were 5.3 pg/mL for CD90 and 1.95 pg/mL for CD83. Based on standard curves run in duplicate on each test plate, CurveExpert Basic Software (version 1.4, Hyams Development) was used for calculation of the sCD90 and sCD83 values.

### 2.3. Data Analysis and Statistics

The data were analyzed using GraphPad Prism (version 8.0.1; GraphPad Software, Inc.; http://www.graphpad.com) statistical software. Statistical significance of difference among mean values was evaluated by the Mann–Whitney *U* rank sum test, one-way ANOVA, or Kruskal-Wallis one-way analysis of variance on ranks. Mean values are presented throughout the text and figures ± the standard deviation (SD). For all analyses, differences were considered statistically significant at *p* ≤ 0.05.

The diagnostic accuracy of the CD90 assay was evaluated by 2 × 2 contingency table of positive and negative results (Table 2) obtained at the proposed cut-off value and the calculation of common metrics, such as sensitivity, specificity, positive predictive value (PPV), negative predictive value (NPV), and overall effectiveness (accuracy) (Table 3).

## 3. Results

### 3.1. Screening Test of Serum CD90 for Diagnostic Significance in Endometriosis

Soluble CD90 molecule was measured in serum samples from healthy controls and was compared to the levels of expression in endometriosis patients. The results show an average level of 334 ± 228 pg/mL for healthy donors (*n* = 28) and 1160 ± 856 pg/mL for endometriosis cases (*n* = 27) (Figure 1(a)). Two healthy controls, which represent an incidence of 7.1% from the group of 28 volunteers, diverged with 957 pg/mL and 1145 pg/mL CD90 serum levels. However, the rest of the samples (92.9%) were distributed homogenously with significantly lower values between 92 and 480 pg/mL. The obtained upper normal value of sCD90 in the group of controls, excluding the outliers, was 479.4 pg/mL. Therefore, a cut-off level was set at 479.4 pg/mL to define low and high content of sCD90 in serum of patients in order to perform a condition-based analysis of the specimens. According to the threshold, 8 out of 27 (~30%) endometriosis patients had sCD90 values in the control range and the rest of the patients had intermediate or high serum sCD90 levels, suggesting a possible stratification of patients. The diagnostic accuracy of the screening test was then evaluated via calculation of sensitivity, specificity, predictive values, and overall effectiveness [43, 44] (Table 3). The test reached 70.4% sensitivity while identifying the patients with the disease and 92.9% specificity of true negative read-outs within the control group. The clinical usefulness of the test was estimated via its predictive power, which showed 90.5% for PPV and 76.5% for NPV and 81.8% diagnostic effectiveness of the test.

The group of endometriosis patients exhibited a clear heterogeneity of CD90 values. Nineteen specimens had high CD90 values, but 8 were similar to controls. Their occurrence raised the hypothesis that there might be an association with the disease evolution and/or the functional phase of menstrual cycle, which are possible variables. To examine this, CD90 results were plotted against the endometriosis stages (I—minimal, *n* = 2; II—mild, *n* = 5; III—moderate, *n* = 11; and IV—severe, *n* = 8). A well-defined clustering of 6 out of 11 cases (54.6%) with low sCD90 was evident within stage III (Figure 1(b)), whereas single cases in stage I and stage II were evident. The investigation of sCD90 in relation to the functional phase of menstrual cycle showed no specific clustering of low values in proliferative (days 1-12), periovulation (days 13-15), or secretory phases (days 16-28) (Figure 1(c)). They seemed evenly distributed and represented 35.7% (proliferative, *n* = 5/14), 22% (periovulation, *n* = 2/9), and 33% (secretory, *n* = 1/3) negative cases in each phase.

Altogether, the results from the test show ~70.4% coincidence of sCD90-positive/high results in serum of patients with endometriosis, while the remaining 30% of patients with sCD90-negative/low results predominantly cluster in stage III of the disease.

### 3.2. Screening Test of Serum CD83 for Diagnostic Significance in Endometriosis

Serum level of sCD83 was investigated in the control (*n* = 30) and endometriosis (*n* = 21) groups of women. The average value in asymptomatic controls was 881.6 ± 251 pg/mL (Figure 2). This distribution was comparable to the endometriosis patients, which had an average of 1043.9 ± 343 pg/mL. Due to the lack of a distinct difference between the groups (*p* = 0.0726), it was concluded that the sCD83 molecule had no diagnostic power for predicting endometriosis.

## 4. Discussion

Endometriosis presents with dysregulation of multiple genes and proteins [45], such as enzymes, metabolites, signaling, and immune molecules [13, 46, 47], some of which are still not elucidated. This initial study for biomarker discovery considered patients with all stages of the disease, in order to search for a marker indicative of the condition as a whole. Since the patients with endometriosis showed a significant elevation of sCD90 when compared to control specimens, we evaluated the power of the sCD90 screening test for possible diagnostic use. Due to the small sample size which did not allow an ROC curve analysis (a comparison of sensitivity against false-positive rate), the threshold value was considered on the basis of highest sensitivity and the minimal false positive cases in the group of healthy women. Consistently, 92.9% of the control subjects clustered in the range 91.9-479.4 pg/mL sCD90, without any visible segregation, whereas two patients had outlying values. We observe that in healthy women, sCD90 is released in blood at background levels (334 ± 228 pg/mL), while asymptomatic disease conditions could be a presumptive reason for elevation of sCD90 molecule in some control women. Therefore, the outliers were discarded from consideration and the highest value (479.4 pg/mL) from the normal distribution of controls was chosen for a threshold in the study. In turn, the endometriosis patients revealed a spectrum of high and low sCD90 values, with a large standard deviation. As the large variation within the group suggested a stratification of the patients, we tried to uncover a correlation between disease progression and sCD90 levels. This examination did not reveal any overall trend of sCD90 values correlating with disease progression, such as a gradual increase though all 4 stages. However, almost all of the low values in endometriosis patients were in stage III. 54.6% of the patients classified in stage III had low sCD90 levels. Possible explanations of this fact could be the heterogeneity of the disease background due to multifactorial causes, changes of inflammatory processes, or an as yet unknown functional transition in stage III due to specificity in disease evolution. Nevertheless, the test showed high statistical power (^∗∗∗∗^*p* < 0.0001) and could specifically distinguish between women with endometriosis and controls. Based on the agreement between the disease condition and the positivity of the test, we suggest that the test should rather be interpreted by the quality of the reaction (“positive” or “negative”) than the quantity of sCD90. In that respect, we consider that the variance in the intensity of sCD90 expression is not that indicative.

Assessing the diagnostic accuracy for the sCD90 test in serum of 55 subjects shows an outcome of 70.4% sensitivity and 92.9% specificity. These results are within the requirements of the minimally acceptable criteria, which some authors define as 70-100% sensitivity and 60-100% specificity [44] and thereby identify sCD90 molecule as a promising biomarker test option. Potentially, the sCD90 serum levels can be recommended as a secondary diagnostic factor for patients with primary findings of sonography, pain, and infertility symptoms and as a primary test for broad screening of female populations [44].

Evidence about the dynamics of sCD90 release in disease conditions is scarce so far. However, a few reports suggest it as a potential biomarker in urine and serum from prostate cancer [48] and systemic sclerosis patients [49]. The source of the sCD90 is not confirmed but some investigations speculate that it originates from fibroblasts and endothelial cells from the affected tissues [26, 28, 49]. A study demonstrates that shedding of sCD90 molecule from cell surface of differentiated myofibroblasts can be mediated by inflammatory (TNF-*α* and IL-1) and fibrogenic (FGF-1 and TGF-*β*) cytokines and thereby leads to its accumulation in culture medium [26]. This finding suggests that aberrant differentiation of cells and/or dysregulated release of factors in pathologies can increase sCD90 in serum of patients. Endometriosis would fit this pattern because it distinctly presents with displaced and abnormal tissue differentiation and chronic pelvic inflammation [13, 15].

The investigation of sCD83 molecule showed no relevance to endometriosis since its serum levels in diseased subjects remained equivalent to controls. Regardless of the nonassociation of sCD83 with the disease, we report the finding as informative, because it adds to the knowledge of which proteins in the blood of patients are unchanged [47].

Currently, medical management of suspected cases of endometriosis is hampered by the lack of noninvasive, fast, reproducible, and affordable diagnostic tools for early and reliable detection of the disease. ELISA tests are in wide clinical use and would be technically highly suitable.

To date, more than 100 molecules [47] in peripheral blood and more than 200 endometrium-related molecules [45] have been reported as putative markers in endometriosis, with variable diagnostic efficiency. At present, the marker discovery for endometriosis is focusing on sequential and epigenetic analyses of genomic and mitochondrial DNA [16], signaling pathways [13], operational glycoproteins, and metabolites, which are involved in inheritance, localization, microenvironment, and endocrine dysregulation of the disease. Combinations of different diagnostic markers and approaches could help in decoding the heterogeneity of endometriosis, which remains a major obstacle to diagnosis.

## 5. Conclusion

CD90 is involved in basic cellular processes that can be malfunctional in pathological conditions. This study shows that increased sCD90 in serum is a specific phenotype that associates with endometriosis. Quantitative evaluation of sCD90 shows over cut-off values in all disease stages but also a tendency of unexplained accumulation of below cut-off values in stage III, suggesting a stratification of the patients. Due to the limited number of patients in this study, further investigation and validation of diagnostic and/or predictive power of sCD90 in serological tests need to be performed. However, the accuracy of sCD90 observed here is comparable to other highly evaluated candidate markers for endometriosis and would seem to indicate considerable potential.

## Figures and Tables

**Figure 1:** The levels of soluble CD90 determined by ELISA in serum samples from (a) healthy (open circles) and endometriosis (black circles) women. The values in the top left corner denote FP (*n* = 2), TP (*n* = 19), TN (*n* = 26), and FN (*n* = 8) cases. (b) Patients in different stages of endometriosis and (c) patients in the functional phases of the menstrual cycle. The red line represents the threshold value set at 479.4 pg/mL. The bars represent mean ± SD. NS: not significant. ^∗∗∗∗^*p* < 0.0001.

**Figure 2:** Circulating sCD83 in human serum of healthy and endometriosis women. The scatter plot represents the levels of sCD83 in picograms per milliliter in human serum of healthy (open circles) and endometriosis (black circles) women determined by ELISA. The bars represent mean ± SD. NS: not significant.

**Table 1:** General characteristics of patients with endometriosis.

Total	*n* = 27
Age (years)^∗^	34.7 (23–46)
Hormone therapy	
Yes	—
No	27
Endometriosis stage	
Stage I	2
Stage II	5
Stage III	11
Stage IV Undefined	8 1
Menstrual phase^+^	
Proliferative phase (days 1-12)	14
Periovulation (days 13-15)	9
Secretory phase (days 16-28)	3
Undetermined	1

^∗^Mean (minimum-maximum value) is presented. ^+^Patients' menstrual status at the time of peripheral blood sample collection.

**Table 2:** The contingency table of a diagnostic accuracy study.

	Actual positive	Anamnesis negative
Predicted positive	True positive (TP)	False positive (FP)
Predicted negative	False negative (FN)	True negative (TN)

**Table 3:** Diagnostic accuracy measures.

Measure	Formula
Sensitivity	TP/(TP + FN)
Specificity	TN/(TN + FP)
PPV	TP/(TP + FP)
NPV	TN/(TN + FN)
Accuracy	(TP + TN)/(TP + FP + TN + FN)

## Data Availability

The results from this study have not been published in archives, databases, or repositories.
